# The Application and Development of Mural Art in Urban Public Environment Landscape Design

**DOI:** 10.1155/2022/3346648

**Published:** 2022-10-11

**Authors:** Weihua Zhou

**Affiliations:** Zhejiang Normal University, Jinhua 321004, China

## Abstract

With the gradual improvement of social and economic levels, cities not only meet people's basic living needs, but also have an artistic expression to a certain extent, and the public pays more attention to the beauty of the external environment. Landscapes in cities are settlement landscapes characterized by man-made landscapes, which are not only a cultural resource but also an ecological environment resource. Murals are also the first works of art of mankind. According to records, murals are the largest number of artworks in China. It is a popular work of art, representing social functions with historical value, aesthetic value, political significance, and educational function. Due to the great influence of the latest technology and emerging technology on urban art concepts, murals are widely used in urban public landscapes in Europe and America. Its grand and strong space coverage, not wasting too much space, and its imperceptible influence on vision make it the main element of urban public art. Therefore, the mural design in the urban public environment can improve China's current urban atmosphere and enhance urban characteristics. Bring the citizens a historical and cultural understanding of the urban environment they live in and enjoy art. According to the interrelationship between the city and the public environment and the human mural art, based on the relevant theoretical knowledge of urban planning and design, urban public art management, and based on the basic characteristics of human mural art, this study combines a large number of domestic and foreign cases, starting from the characteristics of the natural environment and human urban environment. This article studies the relationship between mural design and architectural design concepts and concepts in urban public environment landscape design.

## 1. Introduction

China is an ancient country with a long history and splendid cultural heritage and is also one of the world's historical and cultural centers where tangible and intangible cultures coexist. Among them, the mural can be said to show the natural pictures of ancient and modern human beings, the universe, natural images, and social life, and the so-called murals are painting art on the walls, which is one of the earliest painting activities in human society. In fact, the origin of human mural art can be traced back to the original Stone Age. Beginning with the carving of patterns on stone and ornaments, and gradually developing to painting in spacious caves, the tribes originally recorded the history of their race only in this way. This kind of performance art activity has undergone long development and evolution along with the history of murals, and gradually transformed into a way for ancestors to pursue the beauty of life, which has led to the emergence of “mural” art. Mural paintings are not only a testimony to the use of human beings to transform nature with their own wisdom and tools but also a variety of expressions of spiritual pursuits while constantly possessing rich products. Mural painting is one of the main carriers of inheriting ancient civilization, it is in the form of painting, through the composition of two-dimensional space, the use of various lines and colors to contain civilization, thought and art, known as “museum on the wall”, with high artistic and historical research value.

Public art refers to art forms that are public and serve the public. Based on the social environment and design system level, this study analyzes the landscape problem, takes the public environment and places as the background of the art design, and carries out art design in various public places, reflecting the humanistic care in the works of art. In the 1980s, American architects clearly pointed out that the key to the current development is to let the public form a general recognition of environmental landscape design [1]. After 2000, due to the rapid growth of social culture, artistic activities were also promoted, and various design concepts emerged in endlessly [2]. They regard improving and creating the environment as the focus of their art design [3].

Urban landscape design is a very important part of environmental art, and it is also the finishing touch of the latter [4]. This is because the urban landscape is generally vivid and artistic, which can give the public a more comfortable leisure viewing experience. In the context of rapid social and economic development, the per capita income of residents continues to increase, so that they are no longer satisfied with the richness of material life, but focus on the satisfaction of spiritual life [5]. Therefore, all cities have increased their attention and investment in the urban space environment and paid more attention to the artistic presentation of urban space for public life to meet the aesthetic pursuit of the public [6].

In foreign countries, the origin of modern public art is the Mexican mural movement in the 1920s [7]. With the support of the national government at that time and the cooperation of artists and all walks of life, this activity expressed the culture of the Chinese nation through the murals of urban public buildings, publicized the culture of the Chinese nation, and reflected a strong political concept [8]. Turn performance into an art activity closely related to public life, public environment, and political activities [9]. Mexican painting art has gained a corresponding position in the world, thus forming a wonderful flower in human painting art [10]. After the Second World War, many Western European developed countries adopted innovative methods in considering the urban nature, functional transformation, and the beauty and harmony of urban morphology. Therefore, in the early 1990s, the French redesigned the city with Paris as the center, returning the postindustrial revolution of France to the traditional and romantic urban form. In the late 1970s, France proposed the city of “art in the city”. Construction purpose [11].

The Dunhuang murals of the Tang Dynasty follow the basic tones of the Sui Dynasty in terms of color, the colors are more abundant, and the overall tone is brilliant and bright, complementary and appropriate, showing the beauty of the decoration of the picture. In the entire Tang Dynasty, the murals are more prominent in the richness of the colors and the sense of grandeur, which makes people linger.

We can find that the research and design of public environmental technology in the west is an urban construction mode supported by social and economic forces. It is highly materialized and has entered the consideration range of current social and political behavior to position the cultural life [12]. With the development of China's market economy and the Chinese government's efforts to build a city brand, a civilized city and a harmonious society, do we have similar problems? Figure 1 shows the development trend of modern environmental art in China. There have been many academic papers on the relationship between urban public art and civilization from urban research, cultural communication theory, ecological research, urban anthropology, etc., and the focus and entry point of the articles are mainly focused on contemporary mural art and its participation environment, as well as the humanization and development of Urban Landscape [13]. In the construction of urban regionalization, through the establishment of urban community main services, the historical, cultural, and social functions of public space are investigated, and the relationship between urban regional civilization and citizens is studied [14]. The development prospect of this field in China in recent years will be further theoretically guided, and then the murals in our country will show the possibility of strategic positioning and implementation of cultural, contemporary, and public nature [15]. This study analyzes landscape problems based on the level of social environment and design system, takes the public environment and places as the background of art design, and carries out artistic design in various public places, reflecting the humanistic care in works of art.

## 2. Theoretical Research

### 2.1. Theoretical Overview of Mural Art

#### 2.1.1. The Concept of Murals

Concept and category murals are also known as decorative wall paintings. It is a circle formed on the natural or artificial wall surface by means of color painting, sculpture, and other modeling techniques, focusing on the interior surface of the decorative building [16]. In the early days, people sculpted and painted murals on rocks to replace the original text to explain and record history. Painting became an independent art form in the early days. There are two kinds of existing prehistoric Relics: cave paintings and cliff murals, which have been unearthed in Europe, America, Africa, Oceania, and Southeast Asia [17]. Due to the development of Architectural Science and Technology, Chinese murals also began to gradually transition from cave murals to modern architectural murals [18]. As an important decorative component of architectural design, painting realizes a balance system between the authenticity of architectural design and the infectivity of art through the common adaptation of architectural design and art [19]. It is an important member of art, actively participates in the construction of contemporary cities, and plays an important role in improving the quality of the city and shaping the image of the city [20].

#### 2.1.2. Characteristics of Murals

The advantages of architecture are mainly reflected in its special dependence on architecture, its openness to public space, its diversity of expression forms, and its creation of public space aesthetics. The characteristics of painting depending on the special space environment determine the nature of painting different from pure art sculpture.  Table 1 shows the comparison of different murals. Painting and architectural design together form a whole, which is an organic combination of environmental art. Under the common influence and function of the two, the artistic beauty and the environmental spirit have been reflected and the art has been made public. In urban construction and space environments, attention is paid to the needs of human aesthetics and spiritual life. Therefore, mural art has great openness and popularity in the construction environment. In the past, wall art was one of the few powerful traditional arts in Chinese history. Both modern and contemporary walls have greatly adapted to the public's thinking, attention to people, and people's requirements for spiritual life. The media capabilities of modern murals are more diversified, such as information, ideas, technology, market, which also greatly enrich the expression forms of modern wall art, such as the diversified application of functions, popularization, and high-tech materials.

#### 2.1.3. The Function of Mural

Murals play a practical aesthetic role in the urban spatial landscape. The practical function also includes space guidance—guiding the aesthetic order in the space through the city wall, so that we can experience cohesion in the urban environmental landscape. Spatial recognition: the appearance of modern architectural design has declarative and symbolic visual features. Artistic function, usually a beautiful wall, is not good-looking when placed in a certain position because the function of the wall and the carrier attached to it are inseparable from its position.

### 2.2. Overview of Urban Landscape

#### 2.2.1. The Connotation of Urban Landscape Design

Urban landscape is regarded as an act of urban beautification. Urban landscape covers a wide range, including natural conservation ecology, historical and cultural buildings, so that people living in the city can feel the joy, identity, and beauty of the city. It is proof of the quality of the urban landscape, and the quality of life that is artificially improved through these original urban connotations is the basic concept of the urban landscape.

The city is composed of many buildings, and the outdoor space outside the buildings is often neglected, but these spaces have a great relationship with the quality of the urban landscape. The urban landscape is not only a visual impact, the city Landscape refers to the experience of living in the city, which produces a sense of quality to the place. Therefore, in order to make urban residents have psychological pleasure, identity or beauty, as well as physical comfort and hygiene, urban landscape has a great influence.

#### 2.2.2. Design Principles of Urban Landscape

The scope of urban landscape design covers a wide range, which is not the same as the general design. Starting from the “point”, it refers to the focus of urban space. From the perspective of human vision, it is divided into attention points, landmark points, and nodes. These are the “dots” most often seen in the city. The “line” mainly refers to the axis, which can control the structure of urban space and the running route of people. It is not a real line but an induction line. In the urban landscape, “face” refers to the interface, and “body” refers to the space or volume. The so-called space is the part of “nothingness” that people feel under the limitation of objects. As for the “color” of the urban landscape, it mainly refers to light. Light is another main factor that affects the shape and stimulates the perception. The light source is divided into two parts: natural light and artificial light (see Table 2).

## 3. The Development Trend of Mural Art in Urban Public Environmental Landscape Design

### 3.1. Reflections on the Design and Construction of Chinese Contemporary Urban Public Environment Murals

#### 3.1.1. Urban Resource Culture

The natural geographical environment affects the pattern, functional layout, and urban development appearance of the city. In modern cities, the urban environment closely related to human survival can be divided into the public environment, business environment, and daily life environment.  Table 3 shows the spatial structure layout of different cities. On the contrary, different urban environments and different resources have caused great differences in materials, architectural structures, and artistic styles in various places in human history. “Traditional civilization” refers to the aggregation of various material and spiritual properties provided by people in the human environment, and refers to the synthesis of scientific knowledge, religious belief, literature and art, moral character, social laws and customs, and various phenomena. While urban civilization changes with the development of political system and economic society in the world, and pursues individuality in the process of change. Based on the concept of modern anthropology, the study of urban civilization has also created different forms of living space for people. Politics, culture, belief, legal system, customs, and ethics determine the overall image development and environment of a city. However, modern cities are the further development and sublimation of economic civilization in the new era on the basis of further condensing its traditional cultural content. Therefore, the continuous improvement of the city depends on the civilization created by the previous generation. And history is also the soul of the process of urban development. Although the new mode of production and life requires people to adapt to the needs of society, people must preserve the imprint of our history and civilization.

### 3.2. The Preparatory Stage of Mural Design in Urban Landscape Design

The preparatory stage is the key to the positioning of the content, style, and expression techniques of the murals. Preliminary preparations include the following: 1. Understand the nature, objectives, municipal requirements, and the responsible person of the street community where the mural is to be planned for the project. 2. Understand relevant policies and regulations. 3. Research and investigate the human factors and external factors of the environment, make written materials of design concepts and ideas and find out the corresponding design intentions and creative methods through the survey and photography of the surrounding scenes of the murals. 4. Modification after extensive solicitation of opinions from experts and the public. See Figure 2 for details.

### 3.3. Relevant Factors and Process of Mural Design

Today, mural art has begun to move towards art museums, into the daily life of the people, and become a part of public art by integrating with nature. The means and forms of art should be determined according to the urban geographical environment. In the architectural design, we should consider the use of the artistic expression of murals, and methods of expression, highlighting the characteristics of the urban region, so as to improve the national characteristics of the city.

### 3.4. The Development Trend of Contemporary Urban Murals in China

After entering the twenty-first century, my country has experienced rapid economic development.

In the development of the whole market economy, the construction of urban culture will inevitably lead to the improvement of citizens' spiritual life needs. Building an ecologically civilized city has become a new requirement of all cities in China in the process of economic and social development. However, due to some conditions, in some cities in China today, the appearance of some buildings conflicts with the style of surrounding communities, specifically in the following aspects:

With the continuous expansion of Chinese cities today, the size of the squares has increased, and the division of urban regional functions has increased, making urban life and work faster and faster, such as industrial areas, cultural areas, commercial areas, etc. Media installations are of different colors and locations. It blurs the connection between the spatially oriented environmental form in the city and the architectural language.

The murals of public space in Chinese cities can not only highlight the beauty and connotation of the design of old buildings but also refresh the impact of the design of old buildings on the beauty of the surrounding urban environment. More importantly, it harmonizes the individual buildings and the surrounding urban environment in terms of color and style.  Figure 3 shows the investment of different cities in mural design. It emphasizes the cultural characteristics and spiritual guidance of the undetermined results of urban functional areas, so that the urban landscape carries the corresponding cultural information, thus promoting people's awareness of regional subjects and regional separation of the urban landscape. It improves the order of urban landscape. At the same time, it makes full use of the art techniques of urban murals, which can break through the constraints of traditional venues and improve the size and specification of visual space in the space, improve the coordination between buildings and the environment, and inject art into the visual experience of urban public spaces even in urban commercial centers.

The development trend of urban murals in my country is mainly reflected in the following two aspects: one is the cross-combination of multiple disciplines, not just at the artistic level, but especially the urban function level. Second, urban architecture should develop toward a more comprehensive and unified trend. Establish rich and elegant urban public space and green urban landscape and build the enterprise brand image. Specifically, we must make solid efforts at the following levels:

1. The government advocates urban construction. All functional departments of the government should make overall arrangements for urban murals.
2. Citizens' Participation, administrative personnel, and design personnel should make design adjustments and modify design defects according to the good opinions of citizens. For example, we will extensively listen to residents' suggestions in various forms, such as seminars, special newspapers and periodicals, and television.
3. Technical training for talents: professional training for artistic talents divides the majors of art research institutes into two aspects such as creative practice and academic research.
4. By using enterprises to support art we should advocate using enterprises or organizations to support art and make contributions to improving national culture. This mode is quite common in the operation of companies in European and American countries. First, the company acquires the paintings of artists or donates them to the society or the municipal government. The second is the murals made by the company to create an image or beautify the environment for its own company. If it is in the urban public area, it needs to be reviewed or modified by relevant experts and scholars invited by relevant government departments, and the public's opinions should be consulted. Implement the planned urban mural design.

China's contemporary urban painting is the inheritance and innovation of China's traditional cultural painting. With the vigorous development of modern urban culture, the public aesthetic category of urban space in the future will also be injected, not only the pure political education, pure art education or pure economic category of architectural art. Thus, the full affirmation of the development of urban mural art in China is the spirit of the times embodied in the Chinese national spirit and urban environmental art.

## 4. Countermeasures and Suggestions for the Application of Mural Art in Urban Public Environmental Landscape Design

### 4.1. Audience

#### 4.1.1. Strengthen the Aesthetic Education of the Masses

“The important artistic feature of murals is its aesthetic value…. Murals have not changed their common nature with other types of paintings. They must directly vent their inner emotions through painting materials or by means of craftsmanship to express and grasp the social functions and aesthetics of murals. Values and other deeper pursuits.” Muralists or designers, facing the constraints of various factors and prereading of places and spaces, hope to find the link between the characteristics and lack of public space and the spiritual demands of the public.

For the development of public landscape art design, we should also enhance the audience's aesthetic taste, identify and appreciate art, arouse the public's curiosity about public art and mural design, and care about the beauty around life, which will help us improve the quality of the living environment.

#### 4.1.2. Narrowing the Gap between Urban and Rural Areas

In the context of the continuous development of my country's market economy, the coordinated development of urban and rural areas has also been gradually promoted. It is particularly obvious that the various production bureaus existing between urban and rural areas continue to decrease.  Figure 4 shows the income gap between urban and rural residents in my country. But at the same time, the higher-level needs of urban and rural residents in art and other aspects cannot be effectively met. Official statistics reflect the seriousness of the resource gap between urban and rural areas. Because funding varies from place to place, results are less likely to attract attention, and there is a lack of fair funding allocation, base selection, and establishment mechanisms. The funding for the design of public art or mural art in a city is often the funding for the construction of a primary school in a rural area. For most rural areas, in addition to insufficient funds, they also face a shortage of professional talent resources.

### 4.2. Institutional Aspects

#### 4.2.1. Improvement of Regulations

To a large extent, public policy influences and restricts the creation and development of mural design. According to the “third way” theory put forward by European and American countries, it is known that the interaction between the government and the public should be improved, that is, to a certain extent, the enthusiasm of the public to participate in public cultural activities should be stimulated, and social activities should be used as much as possible. At the same time, the government should also play a guiding role in the process of promoting ceramic art creation, mobilize the enthusiasm of the public to participate, so as to effectively integrate the relationship between various social subjects. If the government can support it from all angles, it will greatly promote the development of public art creation, and it will also help to increase the enthusiasm of artists to create, which in turn will help promote the effective development of public art.  Figure 5 shows the specific process of the simplified urban public environment landscape design. At the same time, the government should also formulate corresponding policies and regulations to effectively promote the development of works of art, and further improve the aesthetic needs of the public, thereby helping to improve the overall appreciation of works of art in society, and will also greatly promote the development of mural design artwork.

#### 4.2.2. Program Simplification

Different departments have different ideas in terms of policy, and often operate independently in terms of implementation. For example, urban design, public art, street furniture in various places have their own achievements in policy results, and lack of cooperation and unity between them has led to the environment becoming increasingly chaotic, and the overall administrative effectiveness is greatly reduced, and the aesthetic value of the city's image is even more impacted. Because of different affiliations, the same base often has inconsistent street furniture and public art, resulting in seriously different views and actions, making the original urban style messier, and too much visual focus will make people tired. Not only will it not produce a sense of beauty, but it will also make people feel oppressed and nervous. Therefore, it is more important to integrate policies. Large-scale planning and design to create unique features and policy views with a sense of unity and order are the most important thinking.  Figure 6 shows the application procedure for urban landscape design.

## 5. Conclusion

In the long-term course of human development, art bears various historical tasks entrusted by history. After the twentieth century, the concept and value of fine arts, as well as the characteristics and meanings embodied in the continuous development process, have also undergone major changes. Adopt various municipal construction measures and legal systems to improve and promote the cultural and artistic level of urban public places and social environment, and maintain a certain artistic taste of the city and the people. This has become an important development strategy and the main content of social welfare measures in the world today. As far as fresco is concerned, it has the following public art status: 1. More emphasis on the expression of personalized thoughts, and comprehensive concern for human aesthetic and spiritual experience; 2. The relationship between the mural content and the urban public landscape. Form a unity, and emphasize the development of urban cultural characteristics in the urban atmosphere; 3. Pay attention to the use of the latest technical materials and technologies to fully reflect the visual and psychological changes caused by the development of science and technology.

## Figures and Tables

**Figure 1:** Development trend of modern environmental art.

**Figure 2:** The preparation process of mural design in urban landscape design.

**Figure 3:** Investment in mural design in different cities.

**Figure 4:** The income gap between urban and rural areas in my country.

**Figure 5:** Simplified urban landscape design process.

**Figure 6:** Urban landscape design application process.

**Table 1:** Comparison of different murals.

Serial number	Tomb owner	Burial age	Age of excavation	Mural content and layout	Remark
1	Li Simo and his wife Yan Tuo	Li Simo was buried in the 21st year of Zhenguan, and Yan Tuo's was buried in the same year	1992	Only the corridors and tombs were cleared. The two walls of Yongdao, “monsters”, “ladies”	Not uncovered

2	Wei Long	The first year of Qianfeng (666)	1991	The two walls of the tomb are painted with “blue dragon” and “white Tiger”	27 pieces were uncovered, now in the Zhaoling museum

3	Li Qin and his wife	Li Qin was buried in the first year of Xianheng, and his wife was buried in the fifth year of Xianqing	1971	The frescoes are completely damaged, and the west wall of the tomb is painted with “six screens”	Not uncovered

**Table 2:** Principles of urban landscape design.

Principle	Describe
Point	Vision is the basic unit that can serve as the center of a pattern basis. In the urban space, the visual focus that can draw people can be divided into the visual center point and the perspective vanishing point

Wire	It is formed by the arrangement of many points along the same direction. It can represent the direction and boundary. The trajectory moved by the points is the line. The expression of the line has many types, including long, short, thick and thin.

Square	When many lines are repeated in the same direction and close together, a surface with an area will be formed. Faces have length and width, but only a tiny height.

**Table 3:** Urban spatial structure layout.

Natural factors		Affect the result	Reason	Example
Terrain	Plain	Most cities are located in the plains	Flat terrain, fertile soil, convenient for farming	Most of our cities are on the third ladder
	Plateau	Cities in the tropics are mostly distributed on the plateau	The tropics are hot in the lowlands and cool in the highlands	Brasilia
	Mountains	Cities are mainly distributed in the middle and low latitudes	The surface is relatively flat with abundant water sources	Fenhe and Weihe valleys

Climate	Suitable climate	Cities are distributed along river valley bottoms or open lowlands	Moderate precipitation, moderate temperature	High proportion of cities in wet areas
	Bad weather	There are few cities in desert areas, alpine areas, and hot and humid areas	Unfavorable precipitation or temperature conditions	There are few cities in the arid regions of northwest my country

River	Water supply	Cities are often distributed along rivers	Cities need a lot of water for domestic and production use	Cities along the Yangtze river
	Transportation	The starting point and ending point of the river can easily form a city	Goods are gathered and transshipped here	Ganzhou
		It is easy to form cities at the confluence of main and tributaries	Mass flow of people and logistics	Yibin, Chongqing, Wuhan
		Where the river bends more	Interchange between river and sea	Shanghai, Guangzhou
	Military defense	Where the river bends more	Defence with natural river surface	Bern, Paris

## Data Availability

The labeled data set used to support the findings of this study is available from the corresponding author upon request.
